The article "Crocus sativus L. Tepal Extract Induces Apoptosis in Human U87 Glioblastoma Cells" was published in 2022. Journal: Biomed Res Int.

# *Crocus sativus* L. Tepal Extract Induces Apoptosis in Human U87 Glioblastoma Cells

**DOI:** 10.1155/2022/4740246

**Published:** 2022-06-10

**Authors:** Shoib Ahmad Baba, Maryam Vahedi, Irfan Ahmad, Bodour S. Rajab, Ahmad O. Babalghith, Safia Irfan, Md. Jamal Hossain

**Affiliations:** ^1^Department of Education, Government of Jammu, And Kashmir, India; ^2^Department of Horticultural Science, Faculty of Agricultural Sciences and Engineering, College of Agriculture and Natural Resources, University of Tehran, Karaj, Iran; ^3^Department of Clinical Laboratory Sciences, College of Applied Medical Sciences, King Khalid University, Abha, Saudi Arabia; ^4^Laboratory Medicine Department, Faculty of Applied Medical Sciences, Umm Al-Qura University, Makkah, Saudi Arabia; ^5^Medical Genetics Department College of Medicine, Umm Al-Qura University, Makkah, Saudi Arabia; ^6^Department of Biosciences, Faculty of Science, Integral University, Lucknow, India; ^7^Department of Pharmacy, State University of Bangladesh, 77 Satmasjid Road, Dhanmondi, Dhaka, Bangladesh

## Abstract

*Crocus sativus* (*C. sativus*) is considered as the costliest spice and an important medicinal plant. Herein, we investigated the effects of tepal extract (TE) of *C. sativus* on the viability of the human glioblastoma cells. Results revealed that TE significantly (*P* < 0.05) inhibited the proliferation of U87 glioblastoma cells in a dose-dependent manner with comparatively lower toxic effects against normal astrocytes. The IC_50_ of TE against U87 glioblastoma cells was found to be 130 *μ*g/mL as compared to 600 *μ*g/mL against normal astrocytes. TE also inhibited the colony formation of U87 cells significantly (*P* < 0.05). The AO/EB and Annexin V/PI staining assays indicated that TE stimulated apoptosis in U87 cells dose dependently. The early and late apoptotic U87 cells increased from 0.66% and 2.3% at control to 14.2% and 21.4% at 260 *μ*g/mL of TE. Moreover, TE caused upregulation of Bax and suppression of Bcl-2. Wound healing assay showed that migration of the U87 cells was suppressed significantly (*P* < 0.05) at 80 *μ*g/mL of TE. Taken together, these results suggest that TE exhibits antiproliferative effects against U87 glioma cells and may prove to be an important source of natural anticancer agents.

## 1. Introduction

*Crocus sativus* L. (*C. sativus*) belonging to family *Iridaceae* is an important medicinal plant [1]. Medicinal properties of *C. sativus* are generally attributed to the presence of a specific group of compounds. These compounds are formed by the oxidative cleavage of carotenoids and are commonly known as apocarotenoids. These apocarotenoids include crocin, safranal, and picrocrocin in considerable quantities [2]. In addition to apocarotenoids, *C. sativus* is also a rich source of flavonoids such as kaempferol, taxifolin, and naringenin, to name a few [3, 4]. *C. sativus* has array of medicinal properties, for instance, antidiabetic, anti-inflammatory, cardioprotective, and anticancer [5]. Samarghandian et al. showed that *C. sativus* extract inhibits pulmonary tumor suppression via activation of apoptosis [6]. Bakshi et al. showed that crocin from *C. sativus* induces apoptosis and cell cycle arrest of the pancreatic cancer cells [7]. In yet another study, D'Alessandro et al. showed that *C. sativus* stigma extract stimulates apoptosis to suppress proliferation of the human prostate cancer cells [8]. Nonetheless, there is little information on the antiproliferative effects of tepal extracts of *C. sativus*. The present study was therefore undertaken to determine the anticancer properties of *C. sativus* tepal extract against the human U87 glioma cells and to unravel the possible underlying molecular mechanisms.

The article "Crocus sativus L. Tepal Extract Induces Apoptosis in Human U87 Glioblastoma Cells" was published in 2022. Journal: Biomed Res Int.

Gliomas are prevalent type of tumors of central nervous system and responsible for significant number of human mortalities [9]. As per the American Brain Tumor Association, gliomas constitute 24.7% of all the primary brain tumors and 74.6% of all malignant tumors [10]. Unfortunately, the survival rate of the glioma patients is very poor. The average survival period of the patients with the currently available treatment strategies is less than 60 months for low-grade glioma and below 15 months for the advanced stage disease [11]. Therefore, there is urgent need to identify efficient treatment strategies for the management and improvement of survival rates of the glioma patients. Consistently, the present study was undertaken to examine the effects of tepal extract (TE) of *C. sativus* against the human glioma cells. This study will form basis for the identification of lead molecules from *C. sativus* for anticancer chemotherapy.

## 2. Materials and Methods

### 2.1. Cell Lines and Culture Conditions

The U87 glioblastoma cells were cultured in DMEM/F12 containing 10% fetal bovine serum in a humidified atmosphere containing 5% CO_2_ at 37°C. Astrocyte growth medium from an AGM-Astrocyte Medium Bullet kit (Lonza) was used for the maintenance of normal human astrocytes.

### 2.2. Preparation of the C. sativus Tepal Extract

The extract was prepared from shade dried tepals (100 g) of *C. sativus* by maceration with ethanol as described previously [12]. The tepal extract (TE) was then filtered and concentrated at 50°C under reduced pressure on a Rotavapor®. The resultant extract was used for further experiments.

The article "Crocus sativus L. Tepal Extract Induces Apoptosis in Human U87 Glioblastoma Cells" was published in 2022. Journal: Biomed Res Int.

### 2.3. Cell Viability Assay

The glioma U87 and the normal astrocytes were added in 96-well plates with of 5 × 10^3^ cells/well. Then, treatment of the cells with different concentrations (0 to 640 *μ*g/L) of TE for 24 h at 37°C was followed. Next, 10 *μ*L of MTT (5 mg/mL) was followed by an additional 4 h incubation at 37°C. Thereafter, DMSO (10%) was used to solubilise the formazan crystals. Finally, OD_570_ was determined by using spectrophotometer to estimate cell viability.

### 2.4. Colony Formation Assay

Around 5000 U87 glioma cells were seeded in 12-well plates and treated with varied concentrations of TE. The plates were incubated for 14 days at 37°C, and the colonies so developed were fixed in paraformaldehyde for 20 minutes, PBS washed, and subjected to staining for with 0.1% crystal violet for 35 minutes. The visible colonies were PBS washed and photographed under a microscope. The colonies were finally counted using the Image J software.

### 2.5. Acridine Orange and Ethidium Bromide (AO/EB) Staining

AO/EB staining was carried out for the detection of apoptosis in U87 glioma cells. Briefly, the U87 cells were seeded in coverslips with 5 × 10^5^/wells and cultured for 24 h at 37°C. Then, the culture medium was replaced with a fresh medium containing different concentrations of TE. The cells were then again incubated at 37°C for 24 h. Subsequently, AO/EB staining of monolayer cells was performed. Finally, the cells were examined under a fluorescence microscope (×200) magnification, and images were captured.

### 2.6. Annexin V/PI Assay

The U87 glioma cells were collected and then suspended in 500 *μ*L of 1X binding buffer. Then, Annexin V-FITC (5 *μ*L) was added to the suspension followed by PI (10 *μ*L) (Annexin V-FITC detection Kit, Beyotime Biotechnology). The cells were mixed evenly and refrigerated at 4°C for 10 min in the dark. Flow cytometer (Accuri C6, Becton-Dickinson, US) was used to detect the apoptotic cells.

### 2.7. Wound Healing Assay

U87 cells were cultured in 6-well plates with density of 1 × 10^5^ cells/wells to confluent monolayers and subsequently subjected to overnight starvation in serum-free media. Wound scratching was done by sterile pipette tips. The plates were washed to remove the debris, treated with TE, and subjected to incubation for 24 h at 37°C. The wound gaps were photographed at 0 and 24 h time intervals to determine cell migration.

### 2.8. Western Blotting Assay

Treated and control U87 cells were subjected to washing with PBS lysed in ice cold lysis buffer. The protein concertation of each sample was determined by Bio-Rad protein Assay kit. Whole-cell lysates (30 *μ*g) were separated by 12% SDS–polyacrylamide gel electrophoresis and subsequently moved to a polyvinylidene difluoride membrane. Afterwards, western blot analysis was used for specific primary antibodies Bax (sc-7480, Santa Cruz, CA, USA), Bcl-2 (sc-23960, Santa Cruz, CA, USA), and Actin (sc-58673, Santa-Cruz, CA, USA). The membranes were washed three times with TBST and incubated for 2 h with appropriate HRP-conjugated secondary antibody anti-rabbit IgG HRP (Cell Signaling Technology, 7074s, 1 : 2000). Signals were visualized by using the Enhanced Chemiluminescence Plus (ECL Plus) detection system (GE Healthcare).

The article "Crocus sativus L. Tepal Extract Induces Apoptosis in Human U87 Glioblastoma Cells" was published in 2022. Journal: Biomed Res Int.

### 2.9. Statistical Analysis

Each experiment was done with three replicates, and data was shown as mean ± SD. Statistical analysis was carried out by using *t*-test through GraphPad prism 7, and *P* < 0.05 indicated statistically significant difference.

## 3. Results

### 3.1. TE Inhibits the Proliferation of Glioblastoma Cells

The effects of TE were evaluated against the U87 glioma and normal human astrocytes by MTT cell viability assay (Figure 1). It was revealed that the viability of U87 cells diminished significantly (*P* < 0.05) in a dose-dependent manner. At 320 *μ*g/mL of the extract, the cell viability was inhibited by 96.5%. However, the antiproliferative effects of TE were milder against the normal astrocytes. The IC_50_ of TE was found to be 130 *μ*g/mL against the U87 cells as comparted to an IC_50_ of 600 *μ*g/mL against the normal astrocytes suggestive of cancer specific antiproliferative effects of TE. Next, the effects of TE were assessed on the colony-forming potential of U87 cells. Results indicated that the colony formation ability of the U87 cells decreased significantly (*P* < 0.05). Compared to control, the colony formation potential of the U87 cells decreased by 85% at 320 *μ*g/mL of TE. These findings clearly suggest the antiproliferative effects of TE against U87 glioblastoma cells.

### 3.2. TE Induces Apoptosis in Glioblastoma Cells

To find out how TE inhibits the proliferation of the U87 cells, AO/EB staining was performed. AO/EB staining revealed apoptosis to be responsible for the inhibition of proliferation by TE. Fluorescence microscopy showed the presence of different types of cells. The bright green color cells indicate the normal viable cells, the yellowish cells represent early apoptotic, orange cells represent late apoptotic, and the red color cells represent the necrotic cells (Figure 2(a)). Next, Annexin V/PI assay was performed to find out the percentage of apoptotic U87 glioblastoma cells at each concentration of TE. The early and late apoptotic U87 cells increased from 0.66% and 2.3% at control to 14.2% and 21.4% at 260 *μ*g/mL of TE respectively (Figure 2(b)). Western blotting revealed that the expression of Bax increased and that of Bcl-2 decreased upon treatment of the U87 cells with TE (Figure 2(c)). These findings indicate that TE stimulates apoptosis in U87 glioblastoma cells.

The article "Crocus sativus L. Tepal Extract Induces Apoptosis in Human U87 Glioblastoma Cells" was published in 2022. Journal: Biomed Res Int.

### 3.3. C. sativus Extract Suppresses the Migration of Glioblastoma Cells

Next, the effects of TE were also assessed on the migration of the U87 glioblastoma cells by wound healing assay. To overrule the antiproliferative effects, lower dosage of TE (80 *μ*g/mL) was used in wound healing assay. The results showed that TE extract significantly (*P* < 0.05) inhibited the migration of the U87 cells (Figure 3).

## 4. Discussion

Plants have served and will continue to serve as an important repository of bioactive compounds [13, 14]. The compounds or their derivatives have been used as drugs or lead molecules for the development of drugs to treat human ailments [15–17]. Several well-known drugs currently used for the treatment of deadly disease have their origin in plants [18]. *C. sativus* is a well-known medicinal plant, and a wide array of pharmacological properties have been attributed to different parts of this plant [5]. Nonetheless, effects of TE have not been evaluated against human glioblastoma cells. Consistently, herein, we report the anticancer effects of TE against the human glioblastoma cells. It was found that TE inhibited the viability of U87 cells more profoundly as compared to the normal astrocytes. This selective inhibition of U87 cells by TE could be attributed to the fact that several signalling pathways show dysregulation in cancer cells [19], and TE extract might modulate any of these pathways. However, more studies are needed to infer the exact mechanism for the selective inhibition of the U87 cells. Our findings are supported by previous finding wherein *C. sativus* extracts have been found to suppress the growth of different cancers such as colorectal cancer [20]. Chryssanthi et al. reported that the extracts of different *Crocus* species exhibit the potential to inhibit the growth of the breast cancer cells [21]. Similarly, Bathaie et al. reported that crocetin from *C. sativus* could inhibit the growth of the human adenocarcinoma gastric cancer growth *in vivo [*22*]*. In yet another study, Mir et al. showed that crocetin beta-d-glucosyl ester from *C. sativus* could inhibit the growth of the breast cancer cells via ER-alpha/HDAC2 axis [23]. Apoptosis is an essential process which eliminates the defective cancerous cells from the body of an organism and helps to maintain homeostasis [24]. In the present study, we found that TE inhibited the proliferation of the U87 cells by inducing apoptosis. However, at IC_50_ of TE, the percentage of both early and late apoptotic cells was 23.78% indicating that apoptosis alone could not been responsible for the antiproliferative effects of TE. Therefore, more research endeavours are needed to identify other molecular routes through which TE exerts its effects. Nonetheless, our results are supported by a previous study wherein Samarghandian et al. showed that *C. sativus* extract induces apoptosis in pulmonary tumor [6]. Next, TE also suppressed the migration of the glioblastoma cells indicating that TE may also exhibit antimetastatic potential given that migration is an initial step in the metastasis of cancer [25]. Although the present study revealed the anticancer potential of TE extract, more studies including *in vivo* studies are needed. Additionally, the active phytochemical constituents of TE extract need to be identified by natural product chemistry approaches.

The article "Crocus sativus L. Tepal Extract Induces Apoptosis in Human U87 Glioblastoma Cells" was published in 2022. Journal: Biomed Res Int.

## 5. Conclusion

Collectively, the results of this study revealed that *C. sativus* tepal extract suppresses the proliferation of human glioblastoma cells via stimulation of apoptosis. Additionally, it could also suppress migration of the glioblastoma cells. These findings suggest that *C. sativus* tepal extract may prove to be an important source of anticancer agents or anticancer lead molecules. However, further research endeavours involving identification, isolation, and mechanism of action of each component of tepal extract are urgently needed.

## Figures and Tables

**Figure 1:** TE suppresses viability of human glioblastoma cells. (a) MTT assay showing the viability of the U87 cells at indicated concentrations of TE. (b) MTT assay depicting the viability of normal astrocytes at indicated concentrations of TE. (c) Colony formation of the U87 cells at indicated concentrations of TE. Data is shown as mean ± SD (^∗^*P* < 0.05).

**Figure 2:** TE induces apoptosis in human glioblastoma cells. (a) AO/EB staining of the U87 cells treated with different concentrations of TE. (b) Annexin V/PI staining showing U87 cells treated with different concentrations of TE. (c) Western blots showing the effect of TE on the expression of Bcl-2 and Bax in U87 cells.

**Figure 3:** TE inhibits the migration of glioblastoma cells. Wound heal assay depicting the effect of TE extract on the migration of the U87 glioblastoma cells. Data is shown as mean ± SD (^∗^*P* < 0.05).

## Data Availability

All data used to support the findings of this study are included within the article.
